# Elevated Substance P Is a Risk Factor for Postoperative Delirium in Patients with Hip Fracture

This article has been retracted.

**DOI:** 10.1155/2022/5320218

**Published:** 2022-03-31

**Authors:** Wenzheng Zhang, Naixia Hu, Ya Zhang, Anying Wang

**Affiliations:** ^1^Department of Joint Sports Medicine, The Affiliated Taian City Centeral Hospital of Qingdao University, 271000 Taian, China; ^2^Neurointensive Care Unit, The Second Affiliated Hospital of Shandong First Medical University, 271000 Taian, China; ^3^Department of Pathology, The Second Affiliated Hospital of Shandong First Medical University, 271000 Taian, China; ^4^Department of Orthopedics, The Second Affiliated Hospital of Shandong First Medical University, 271000 Taian, China

## Abstract

**Objective:**

Hip fractures are quite common worldwide, especially among the elderly, and are associated with a high incidence of postoperative delirium, which worsens functional results and increases death. The causes of postoperative delirium in patients with hip fractures are unknown, and a separate pathobiology has been hypothesized. Substance P is a neuropeptide that has been linked to a number of immune-inflammatory and neurological conditions. The purpose of this study was to see if serum substance P levels could predict postoperative delirium in a group of hip fracture patients.

**Methods:**

A total of 148 hip fracture patients were enrolled in the study, all of whom had no substantial pre-existing medical or cognitive issues. Demographic and regular laboratory data were gathered as a starting point. ELISA was used to examine substance P levels before and after surgery (after 1 day). Patients were then divided into two groups: “postoperative delirium” and “no postoperative delirium.” Intergroup comparisons, study of delirium prevalence rates in postoperative serum substance P quartile categories, and binary logistic regression for postoperative delirium category as outcome were all done.

**Results:**

Except for serum low-density lipoprotein (LDL) levels, there were no statistically significant variations in preoperative substance P levels or other baseline characteristics between the two groups. The “postoperative delirium” group had significantly higher postoperative substance P levels than the “no postoperative delirium” group (46.36.1 versus 31.94.7 pg/ml). There was a significant difference in postoperative delirium rates between the quartile categories of postoperative substance P, with the fourth quartile having the highest rate. Regression analysis revealed that postoperative substance P levels were related with a significantly increased OR (1.265, CI: 1.172-1.283) of postoperative delirium.

**Conclusion:**

In the current sample of hip fracture patients, a higher postoperative serum substance P level was linked to a higher risk of postoperative delirium. Further research into the utility of early postoperative serum substance P as a delirium indicator in hip fracture patients is needed.

## 1. Introduction

Hip fracture is highly prevalent globally [1–3], particularly among elderly populations, with older females bearing the highest risk [4, 5]. Although declining rates of hip fracture have been reported in several high-income countries [6, 7], it is estimated that global demographic shifts will lead to further increase in hip fracture cases, especially among Asian populations [8]. The projected global burden of hip fracture ranges between approximately 7-21 million by 2050, largely owing to increased life expectancy [9]. Specific risk factors of hip fracture include older age, female gender, low bone mineral density due to osteoporosis or osteopenia, physical inactivity, smoking, high or low BMI, drug, and dietary variables, among others [10, 11]. Delirium is an acute state of confusion and impaired consciousness frequently occurring in hospitalized or severely ill patients [12]. The reported prevalence of delirium in hip fracture patients is high, ranging as high as 20-50% in certain cohorts [13, 14]. Increasing age, institutionalization, pre-existing dementia, and severe illness are among significant risk factors for delirium after hip fracture [14, 15]. Patients who experience delirium after hip fracture at increased risk of short- and long-term adverse outcomes including prolonged hospital stay, ICU admission, medical complications, functional impairment, higher mortality, and incident dementia [14, 16] impose tremendous health-care burden and distress. These findings highlight the potential value of preventive strategies to prevent delirium in this group of patients. At the same time, the present understanding of delirium pathobiology remains inadequate [17], and it has been purported that the pathogenesis and clinical course of delirium after hip fracture may differ from that in medically ill patients [18].

Recent evidence indicates that immune-inflammatory and oxidative stress deregulation arising from an aseptic inflammatory cascade may underlie postoperative delirium after hip fracture [19]. The identification of high-value predictive biomarkers of delirium after hip fracture could enable early identification of high-risk patients for tailored approaches for its prevention. The neuropeptide substance P is widely distributed in the central nervous system and is linked to neural inflammatory processes via increased microvascular permeability in several neurological disorders including traumatic brain injury schizophrenia, stroke, and dementias [20–23]. Thus, the current clinical study was aimed at examining substance P as a predictive biomarker of postoperative delirium after hip fracture.

## 2. Materials and Methods

### 2.1. Ethical Approval

The study protocol was preapproved by the Ethical committee of the hospital, and all study procedures were in accordance with the declaration of Helsinki. All subjects or their legal guardians provided signed written informed consent prior to participation.

### 2.2. Study Population

The present study was designed as an observational study. A total of 261 patients with hip fracture patients among patients were registered, among which 148 patients were recruited for participation in the present study. The inclusion criteria were as follows: (1) definitely diagnosed as hip fracture, (2) meeting standard surgical indications and the patient or family members consenting for surgical treatment, and (3) absence of tumors, autoimmune diseases, or other serious organic diseases. The exclusion criteria were as follows: (1) refusal to participate in the present study, (2) refusal of surgery or no indication for surgery, (3) transfer to another hospital for continuation of treatment, (4) patients with pre-existing delirium before surgery, and (5) pre-existing dementia, tumor, or serious medical illness including heart, liver, lung, or kidney disease. The flow diagram of the study is shown in Figure 1.

### 2.3. Baseline Clinical and Laboratory Data

Once enrolled, participants were assessed for delirium daily before surgery until they were discharged using the Confusion Assessment Method (CAM). The examining doctors or nurses conducted approximately 20-minute interviews with the participants, combined with information from relatives, and scored the CAM. Based on the presence or absence of postoperative delirium, patients with hip fracture were divided into a delirium group and a delirium-free group. After enrollment, the patient's clinical baseline characteristics were collected, including age, gender, and low-density lipoprotein (LDL); high-density lipoprotein (HDL); fasting blood glucose (FBG); glycosylated hemoglobin type A1c (HbA1c); and white blood cells (WBC), neutrophil, and lymphocyte counts.

### 2.4. Sampling and Biochemical Analysis of Serum Substance P Levels

Fasting venous blood was collected early in the morning from the two groups of patients one day before (preoperative) and one day after (postoperative) surgery. The samples were sent directly to the central laboratory on dry ice for analysis or stored at -80°C. The level of serum substance P was analyzed using enzyme-linked immunosorbent assay (ELISA), where the substance P reagent was purchased from a commercial company (Abcam, Cambridge, MA, USA).

### 2.5. Statistical Analysis

Descriptive data with normal distribution was summarized as the mean ± standard deviation, and the categorical data was expressed as the frequency. The *t* test was used for comparison between the two groups, and the nonparametric test was used for analysis of categorical data. Postoperative serum substance P was categorized into quartiles, the subjects were divided into 4 groups in accordance, and the prevalence of delirium in each category was analyzed. Binary logistic regression analysis was used to explore the independent predictors of delirium. In the model, age, gender, and baseline laboratory parameters including LDL, HDL, FBG, HbAlc, WBC, neutrophil, lymphocyte counts, and preoperative substance P were entered as independent variables in the regression model. A *p* value <0.05 was considered statistically significant. All statistical analyses were performed using SPSS 22.0 (SPSS, Chicago, IL, USA).

## 3. Results

### 3.1. Baseline Characteristics and Serum Substance P Levels

A total of 148 patients with hip fractures provided complete data, and based on the presence or absence of delirium, 91 patients were grouped into the “no postoperative delirium group,” whereas 57 patients were grouped into the “postoperative delirium group.” The clinical and laboratory characteristics of these patients (age, gender, HDL, FBG, HbA1c, WBC, neutrophil, and lymphocyte) were not statistically significant between the two groups (*p* > 0.05), while ELISA assays showed that there was no statistically significant difference in the preoperative substance P between the two groups (*p* > 0.05) (Table 1). The baseline LDL levels of the “no postoperative delirium group” (2.4 ± 0.3 mmol/L) and the “postoperative delirium group” (2.5 ± 0.2 mmol/L) were significantly statistically different (*p* = 0.028), while after surgery, the postoperative substance P levels of the “no postoperative delirium group” (31.9 ± 4.7 mmol/L) was found to be significantly lower (*p* < 0.001) than that of the “postoperative delirium group” (46.3 ± 6.1 mmol/L) (Figure 2).

### 3.2. Association of Postoperative Serum Substance P and Risk for Delirium

The prevalence rates of delirium in quartile categories of postoperative serum substance P is shown in Table 2. The prevalence of postoperative delirium showed highly significant variations (*p* < 0.001), with increasing rates of prevalence in sequentially higher quartiles of serum substance P.

### 3.3. Logistic Regression Analysis of Independent Risk Factors for Postoperative Delirium

Binary logistic regression analysis showed that postoperative serum substance P was an independent predictor of postoperative delirium (*β* = 0.175, *p* = 0.033). No significant causal relationship between postoperative delirium and other baseline characteristics was noted (*p* > 0.05) (Table 3).

## 4. Discussion

The present observational study assessed the predictive value of serum substance P as a biomarker of postoperative delirium among 148 patients operated for hip fracture. The key finding of the study was that postoperative substance P levels at one day after surgery were an independent predictor of delirium occurring during the hospitalization period. As compared to those in the first quartile of postoperative substance P, those in the fourth quartile showed twice the rate of delirium during hospitalization (10% versus 20%). Significantly higher odds of delirium (1.265, CI: 1.172-1.283) were noted for each unit increase in postoperative substance P levels, while notably, no relationship was evident between the occurrence of delirium and preoperative substance P levels. Substance P is a neuroregulator from the tachykinin family that is primarily secreted by neural cells along with some immune cells and serves as a key mediator between the neural and immunological systems [24]. High postoperative serum substance P has independently associated with high postoperative pain scores after total knee replacement [25] and rotator cuff repair surgery [26]. Raised serum substance P levels after traumatic brain injury and cerebral hemorrhage are also associated with worse functional outcomes and higher mortality [20, 26–28]. While substance P is primarily secreted by sensory neurons, its biological activities are mediated via its interaction with neurokinin receptors (NKRs), primarily NKR1 [29], which leads to a proinflammatory mediator cascade [24]. Genetic polymorphisms leading to differences in the expression of NKR1 have been documented [30] which may explain the well-recognized variation in circulating substance P levels of both health and diseased states [31].

In the current cohort, the patients presenting with higher levels of postoperative serum substance P plausibly represent a subset of individuals at increased risk of worse immune-inflammatory sequelae in postoperative phase after hip fracture. In an observational study of delirium after hip fracture, a specific cause was identifiable only in 3% of the patients [18], and authors suggested that additional factors such as pain levels or type of anesthesia should be investigated as susceptibility factors. Notably, higher substance P levels are implicated in mediating postoperative pain [25]. In a similar phenomenon, postoperative subjects who manifested increase in substance P levels were found at higher risk for nausea and vomiting as opposed to those whose substance P levels remained unchanged or decreased postoperatively [32]. Although the present study design excluded patients with obvious precipitating factors for postoperative delirium including serious medical illness and pre-existing dementia, incident delirium was noted in 38.5% (57/148 subjects), and only LDL levels were found to be significantly different between the groups, pointing to the role of other unidentified and genetic predisposing factors. While specific molecular mechanisms that may underlie the inter-subject variability in the postoperative Substance P level responses warrant further investigation, the present data strongly suggest that high early postoperative substance P level is a valuable biomarker to identify hip fracture patients at higher risk of delirium. Large-scale studies are essential to identify the optimal cut-off values, specificity, and sensitivity of substance P levels that are clinical relevant, in order to facilitate its clinical translation as biomarker of delirium in hip fracture.

The present findings also suggest to a potential role of NK1 receptor antagonists in the preventive management of delirium in postoperative hip fracture patients. The role of NK1 receptor antagonists has been documented in the prevention of postoperative nausea, emesis, and postoperative pain [33, 34]. NK1 and substance P antagonist agents have also been utilized to improve outcomes after traumatic brain injury, particularly when administered in the early postoperative phase [35–37] and found to decrease postinjury cerebral edema by increasing the blood-brain barrier [38]. It may be hypothesized on the basis of the current findings that similar neuroprotection against postoperative delirium in hip fracture could possibly be achieved by the use of NK1 receptor/substance P antagonist agents in the early postoperative phase.

However, the present findings must be viewed considering the limitations of the current study, which include a modest sample size, no dynamic detection of changes in substance P, restricted inclusion criteria, lack of information about additional potential risk factors for postoperative dementia such as method of anesthesia, and laboratory variables like thyroid or albumin levels [39]. In addition, the regression model did not analyze potential interaction effects between the predictive variables, and clinically significant cut-off values for substance P levels were not ascertained. Considering these facts, the present findings must be considered as preliminary data that highlight the potential of substance P as a biomarker of delirium in postoperative hip fracture patients and also suggest the potential role of its blockade in prevention of this devastating complication.

## 5. Conclusion

In sum, the present observational study demonstrated that higher postoperative serum substance P levels one day after surgery in hip fracture patients significantly increased the odds of delirium during the hospitalization period. These data suggest a that substance P and its antagonists may represent clinically valuable entities for translation towards risk stratification, early diagnosis, prevention, and treatment of postoperative dementia in hip fracture patients and therefore merit further investigation.

## Figures and Tables

**Figure 1:** Flow diagram of the study.

**Figure 2:** The LDL and serum substance P levels in different groups. Compared to no delirium group, ∗*p* < 0.05.

**Table 1:** Characteristics of hip fracture patients with and without postoperative delirium.

	No postoperative delirium (*n* = 91)	Postoperative delirium (*n* = 57)	*p* values
Age (years)	68.6 ± 7.7	68.8 ± 8.3	0.882
Gender, male/female	60/31	39/18	0.754
LDL (mmol/L)	2.4 ± 0.3	2.5 ± 0.2	0.028∗
HD L(mmol/L)	1.2 ± 0.3	1.2 ± 0.4	1.000
FBG (mmol/L)	6.7 ± 0.9	6.8 ± 0.8	0.494
HbAlc (%)	6.1 ± 0.6	6.0 ± 0.7	0.357
WBC (×10^9^/L)	7.3 ± 1.4	7.4 ± 1.6	0.690
Neutrophil (×10^9^/L)	5.2 ± 1.5	5.1 ± 1.7	0.708
Lymphocyte (×10^9^/L)	1.8 ± 0.8	1.9 ± 0.9	0.482
Preoperative substance P (pg/ml)	23.6 ± 2.1	23.8 ± 2.5	0.601
Postoperative substance P (pg/ml)	31.9 ± 4.7	46.3 ± 6.1	<0.001∗∗

LDL: low-density lipoprotein; HDL: high-density lipoprotein; FBG: fasting blood glucose; HbA1c: glycosylated hemoglobin type A1c; WBC: white blood cells. ∗*p* < 0.05, ∗∗*p* < 0.001.

**Table 2:** Prevalence of delirium in quartile categories of postoperative substance P levels.

Variable	Q1	Q2	Q3	Q4	*p* values
Delirium, *n* (%)	10 (27.03)	12 (32.43)	15 (40.54)	20 (54.05)	<0.001

**Table 3:** Binary logistic regression of risk for postoperative delirium.

	Regression coefficient	*p* values	OR	95% CI
Age	0.109	0.215	1.062	0.941-1.093
Gender	0.076	0.380	1.051	0.926-1.079
LDL	0.142	0.097	1.083	0.964-1.192
HD L	-0.153	0.136	0.745	0.427-1.081
FBG	0.210	0.233	1.078	0.943-1.190
HbAlc	0.231	0.372	1.064	0.929-1.177
WBC	0.137	0.128	1.146	0.995-1.264
Neutrophil	0.158	0.089	1.067	0.942-1.185
Lymphocyte	0.104	0.241	1.099	0.978-1.136
Preoperative substance P	0.136	0.324	1.050	0.927-1.071
Postoperative substance P	0.175	0.033∗	1.265	1.172-1.283

LDL: low-density lipoprotein; HDL: high-density lipoprotein; FBG: fasting blood glucose; HbA1c: glycosylated hemoglobin type A1c; WBC: white blood cells. ∗*p* < 0.05, ∗∗*p* < 0.001.

## Data Availability

The data utilized which corroborated this study's conclusions are accessible once requested from the corresponding author.
